# Alcohol drinking alters stress response to predator odor via BNST kappa opioid receptor signaling in male mice

This article has been retracted.

**DOI:** 10.7554/eLife.59709

**Published:** 2020-07-21

**Authors:** Lara S Hwa, Sofia Neira, Meghan E Flanigan, Christina M Stanhope, Melanie M Pina, Dipanwita Pati, Olivia J Hon, Waylin Yu, Emily Kokush, Rachel Calloway, Kristen Boyt, Thomas L Kash

**Affiliations:** Bowles Center for Alcohol Studies, Department of Pharmacology, University of North CarolinaChapel HillUnited States; University of CalgaryCanada; University of California, Los AngelesUnited States

**Keywords:** alcohol, stress, predator odor, dynorphin, kappa opioid receptor, norBNI, Mouse

## Abstract

Maladaptive responses to stress are a hallmark of alcohol use disorder, but the mechanisms that underlie this are not well characterized. Here, we show that kappa opioid receptor signaling in the bed nucleus of the stria terminalis (BNST) is a critical molecular substrate underlying abnormal stress responses to predator odor following heavy alcohol drinking. Exposure to predator odor during protracted withdrawal from intermittent alcohol drinking resulted in enhanced prefrontal cortex (PFC)-driven excitation of prodynorphin-containing neurons in the BNST. Furthermore, deletion of prodynorphin in the BNST and chemogenetic inhibition of the PFC-BNST pathway restored abnormal responses to predator odor in alcohol-exposed mice. These findings suggest that increased corticolimbic drive may promote abnormal stress behavioral responses to predator odor during protracted withdrawal. Various nodes of this PFC-BNST dynorphin-related circuit may serve as potential targets for potential therapeutic mediation as well as biomarkers of negative responses to stress following heavy alcohol drinking.

## eLife digest

The connection between stress and alcohol use is highly complex. On one hand, there is the idea of having a drink to ‘steady the nerves’. On the other hand, in alcoholics, abnormal responses to stress often accompany heavy drinking. In this case, it remains unknown whether stress cause excessive drinking, or vice versa.

Areas of the brain that normally help respond to stress work differently in long-term, heavy drinkers. One example is a structure called the bed nucleus of the stria terminalis (BNST), which is over-active in anxiety disorders and is also associated with some of the symptoms of alcohol withdrawal. The mechanism behind both problems is thought to be a specific ‘signaling system’ that is activated by a small molecule called dynorphin.

Previous research into the effects of dynorphin was performed either in the context of alcoholism or of anxiety disorders, but it was not known if there was a connection between the two. Therefore, Hwa et al. wanted to determine how prolonged alcohol use might affect responses to stress, and whether dynorphin signaling plays a role.

To model long-term alcohol use in the laboratory, a group of mice was given free access to alcohol every other day, ensuring that they developed the mouse equivalent of a drinking habit. After six weeks, these ‘heavy drinkers’ went through a period of abstinence, mimicking alcohol withdrawal. Then, the mice were stressed by exposing them to a chemical that smelled like a fox, one of the mice’s predators in the wild.

When mice smell predators, they normally respond by fleeing from the area and digging up debris to defend itself. As expected, the control mice in this study, which did not drink alcohol, did just that. In contrast, the heavy drinkers largely ignored the predator scent by not digging and even spent time hanging around the area that smelled like the predator. Blocking dynorphin-induced signaling in the alcoholic mice, either using a drug or by deleting the gene that codes for dynorphin, reset the stress response to normal, allowing these mice to avoid the predator and dig as normal. Furthermore, measuring the electrical activity in the brain revealed that the BNST was abnormally active in alcohol-drinking mice, driven by signals from another part of the brain, the prefrontal cortex. This reveals part of the circuitry in the brain responsible for the connection between alcohol withdrawal and the stress response.

These results shed new light on the biological mechanisms underpinning the relationship between alcohol use and stress. In the future, these could be used to determine why heavy drinking can overlap with anxiety disorders, or to develop new treatments that would help recovering alcoholics cope better with stress.

## Introduction

Alcohol abuse exacts a tremendous toll on society, and long-term drinking can dysregulate stress systems in the brain. Prolonged alcohol drinking and withdrawal experiences result in enhanced responsiveness and behavioral sensitivity to stress during protracted abstinence (Heilig et al., 2010). Reciprocally, clinical studies show that negative stress coping is predictive of higher levels of drinking in alcoholics (Noone et al., 1999). As blunted responses to stress have been identified in alcohol-dependent people (Sinha et al., 2011), it is essential to consider mechanisms by which alcohol drinking impacts stress responses during protracted abstinence. While many studies have utilized animal models to investigate how stress drives increased alcohol drinking behaviors (Becker et al., 2011; Gilpin and Weiner, 2017), few have explored the effects of alcohol drinking on subsequent stress responsivity.

Chronic alcohol exposure engages brain stress signaling systems that influence drinking behaviors in a dynamic and complex manner (Koob and Kreek, 2007). One such stress system is the neuropeptide prodynorphin (Pdyn) and its receptor, the kappa opioid receptor (KOR), which has been studied in the contexts of both mood and alcohol use disorders (Lutz and Kieffer, 2013). Limbic structures implicated in alcohol and stress behaviors, such as the bed nucleus of the stria terminalis (BNST), are rich in Pdyn and KOR (Le Merrer et al., 2009). The BNST is an integrative hub that may mediate the negative affective state associated with chronic alcohol use and withdrawal (Koob, 2009; Kash, 2012). KORs throughout the extended amygdala and the BNST alter anxiety-like behavior in mice (Bruchas et al., 2009; Crowley et al., 2016) and mediate stress-induced reinstatement for alcohol reinforcement (Lê et al., 2018).

In this study, we tested whether BNST KOR/Pdyn signaling regulates abnormal stress responses after long-term alcohol drinking. We employed the ethologically relevant predator odor trimethylthiazoline (TMT) as a stressor, which is a compound isolated from fox feces. In rats and C57BL/6J mice, TMT activates specific brain regions involved in stress, anxiety, and fear, including the BNST (Day et al., 2004; Asok et al., 2013; Janitzky et al., 2015), and inactivation of the BNST blocks TMT-induced freezing (Fendt et al., 2003). Recent work suggests that distinct neuropeptide circuits in the BNST may drive opposing emotional states (Giardino et al., 2018), which may be dependent on inputs from cortical sites to affect stress coping behaviors (Johnson et al., 2019). The current series of experiments investigate whether Pdyn neurons and KOR signaling in the BNST can modulate behavioral responses to stress in alcohol-exposed animals. We show that dysregulation of cortical inputs to BNST Pdyn neurons and BNST Pdyn neurons themselves underlie lasting behavioral changes to stressors that emerge after chronic drinking. This is a critical area of study, as mitigating stress responses can contribute to improved alcohol relapse outcomes.

## Results

Male C57BL/6J mice were given 6 weeks of intermittent access to alcohol (EtOH), a protocol known to induce heavy voluntary drinking (Hwa et al., 2011), before behavioral testing during protracted (7–10 days) abstinence [Figure 1A]. Mice consumed high amounts of EtOH [Figure 1B] and increased their EtOH preference over time [Figure 1C]. Further, mice achieved greater than 80 mg/dl blood EtOH concentrations, indicative of intoxication, which correlated with drinking behavior [Figure 1D; R^2^ = 0.59, p=0.0036]. To test stress responsivity during protracted abstinence from EtOH, mice were exposed to the predator odor TMT in the home cage (Hwa et al., 2019). Both water (H_2_O)-drinking controls and EtOH drinking mice showed a TMT-induced increase in plasma corticosterone [Figure 1E; TMT main effect: F_1,10_=26.79, p=0.0004, H_2_O BL vs TMT t_10_ = 3.32, p=0.0154, EtOH BL vs TMT t_10_ = 3.99, p=0.005]. We tracked the location of the mouse relative to the TMT and measured the time spent contacting the TMT and in the far corners [Figure 1F]. EtOH-drinking mice displayed reduced avoidance of the TMT compared to the water (H_2_O)-drinking controls during protracted abstinence [Figure 1G–H]. As an initial screen to identify altered behavior separate from avoidance, we examined stress-related and exploratory behavior in three mice per condition on a second-by-second basis [Figure 1—figure supplement 1]. Since the primary difference among stress-related activities was burying, we focused our further analyses on this typical behavior in response to noxious stimuli (Hwa et al., 2019). Specifically, EtOH drinkers demonstrated reduced burying behavior compared to controls [Figure 1I].

**Figure 1.** KOR regulation of responses to TMT predator odor after long-term alcohol drinking. (**A**) Experimental protocol for 5 mg/kg i.p. KOR antagonist manipulation of predator odor behavior after intermittent EtOH. (**B**) EtOH drinking (g/kg/24 hr) and **C**) EtOH preference/24 hr of male C57BL/6J mice (n = 46 mice). (**D**) Blood EtOH concentrations (mg/dl) correlated with EtOH intake (g/kg/2 hr) in a subset of mice. (**E**) Plasma corticosterone (ng/dl) response 30 min after TMT exposure. (**F**) Representative heatmaps of individual H_2_O (left) and EtOH (right) spatial location in the 10 min test. The circle indicates TMT location. Red color indicates maximum time spent. Aqua color indicates minimum time spent. Pretreatment with norBNI affected: (**G**) TMT contact (sec), (**H**) Time spent in the far corners (sec), and (**I**) Burying (sec). *p<0.05, **p<0.01.

**Figure 1—figure supplement 1.** Home cage TMT predator odor ethograms. Stress-related and exploratory behaviors were observed and plotted using BORIS behavioral software: burying (purple), freezing (brown), grooming (orange), rearing (red), stretch-attend (green), and walking (blue). H_2_O mice are in aqua on the left. EtOH mice are in red on the right. Saline-injected mice are the top plots over the 5 mg/kg norBNI-injected mice on the bottom. Ticks represent time and duration of behaviors during a 10 min test.

**Figure 1—figure supplement 2.** Elevated plus maze and peanut oil tests after intermittent EtOH during protracted withdrawal. (**A**) Schematic of elevated plus maze (EPM) and home cage peanut oil trial after 6 weeks of EtOH exposure, where time (s) spent in the (**B**) open arms and (**C**) closed arms was assessed. (**D**) Representative heat maps of H_2_O and EtOH mice with peanut oil in the home cage. (**E**) Contact with the peanut oil and (**F**) time in the far corners. *p<0.05.

At this protracted time point, another group of C57BL/6J male mice was tested in the elevated plus maze [Figure 1—figure supplement 2A]. EtOH mice showed reduced time spent in the open arms of the elevated plus maze [Figure 1—figure supplement 2B; t_18_ = 2.81, p=0.0115] and equal time in the closed arms as controls [Figure 1—figure supplement 2C]. It is possible that the difference in response to TMT was driven by a change in olfaction. To determine whether olfaction was intact in the EtOH mice, peanut oil was tested as an alternative, appetitive odor. EtOH and H_2_O mice spent similar amounts of time contacting the peanut oil [Figure 1—figure supplement 2D–E] and in the far corners [Figure 1—figure supplement 2F].

Previous studies have shown that activation of the Pdyn/KOR system can modulate stress-induced EtOH seeking (Lê et al., 2018), so we tested if KOR blockade could alter drinking-induced stress behavior. Systemic treatment with 5 mg/kg of the long-acting KOR antagonist norBNI 16 hr prior to TMT exposure reduced EtOH-induced increases in TMT contact compared to saline-injected EtOH mice [Figure 1G; Drug main effect F_1,35_=5.45, p=0.0254, EtOH main effect F_1,35_=15.80, p=0.0003; saline H_2_O vs EtOH t_35_ = 2.95, p=0.0113; EtOH saline vs norBNI t_35_ = 4.12, p=0.0004]. NorBNI also alleviated reductions in burying behavior in EtOH mice compared to saline-injected EtOH drinkers [Figure 1I; interaction F_1,35_=9.70, p=0.0037; saline H_2_O vs saline EtOH t_35_ = 4.52, p=0.0001; EtOH saline vs norBNI t_35_ = 2.47, p=0.0367]. Sample ethograms depict changes in burying behavior in the EtOH norBNI group compared to EtOH saline controls and identify other behaviors mice were engaged in during this test such as rearing, walking, and freezing [Figure 1—figure supplement 1]. Given the potential therapeutic relevance of targeting the protracted time point, we next focused on identifying the mechanism for this long-lasting adaptation in the brain’s dynorphin system.

The BNST is a brain site known for its involvement in stress, anxiety, and addiction, and is regulated by the Pdyn/KOR system (Crowley et al., 2016). Previous studies in rats have shown that TMT increases BNST activity using c-Fos as a marker for active neuronal populations (Day et al., 2004; Asok et al., 2013), so we examined this in a line of *Pdyn*-IRES-Cre x Rosa26-flox-stop-L10-GFP (Pdyn-GFP) mice (Al-Hasani et al., 2015) after intermittent EtOH or H_2_O consumption [Figure 2A]. TMT elicited robust dorsal BNST c-Fos immunostaining, which was greater in EtOH mice compared to H_2_O mice [Figure 2B–C; interaction F_1,23_=12.45, p=0.0018; H_2_O non-stress (NS) vs TMT t_23_ = 6.51, p<0.0001; EtOH NS vs TMT t_23_ = 10.13, p<0.0001; TMT H_2_O vs TMT EtOH t_23_ = 3.92, p=0.0041]. Furthermore, TMT increased expression of Pdyn GFP-expressing neurons in the BNST versus non-stressed (NS) mice [Figure 2D; TMT main effect F_1,23_=4.56, p=0.0437]. Importantly, colocalization of c-Fos in Pdyn-containing cells (BNST^PDYN^) was largest in the stressed EtOH group [Figure 2E; interaction F_1,23_=5.91, p=0.0233; EtOH NS vs TMT t_23_ = 4.66, p=0.0007; TMT H_2_O vs TMT EtOH t_23_ = 3.65, p=0.0081], suggesting an interaction between EtOH, Pdyn, and predator odor stress in the BNST. To determine whether EtOH history affected Pdyn/KOR expression in the BNST, a group of C57BL/6J mice underwent EtOH or H_2_O drinking and were exposed to TMT predator odor before the BNST was taken for fluorescent in situ hybridization with *Pdyn* and *Oprk1* probes [Figure 2F]. Pdyn expression was heightened in the EtOH group compared to H_2_O group [Fig G-H, Pdyn intensity: t_10_ = 2.99, p=0.0136; Figure 2I, Pdyn counts: t_10_ = 2.21, p=0.0512], but Oprk1 expression was not altered [Figure 2J].

**Figure 2.** BNST as a critical site for prodynorphin neurons activated after stress during protracted withdrawal from alcohol. (**A**) Schematic of obtaining BNST tissue for c-Fos immunohistochemistry 90 min post-TMT in Pdyn-GFP mice. (**B**) Representative images of Pdyn (green) and c-Fos Cy3 immunostaining (pseudocolored purple) in H_2_O (n = 8), EtOH (n = 8), H_2_O + TMT (n = 7), and EtOH + TMT (n = 4) conditions. Scale bar is 200 µm. cp = caudate putamen, ac = anterior commissure, Lat sep = lateral septum. (**C**) BNST c-Fos quantification (mm^2^). Aqua bars are H_2_O, red bars are EtOH. (**D**) Pdyn-GFP quantification (mm^2^). (**E**) Colocalization between c-Fos and Pdyn-GFP (mm^2^). (**F**) Schematic of obtaining BNST tissue for in situ hybridization 30 min post-TMT in C57BL/6J mice. (**G**) BNST images of *Pdyn* (pseudocolored red) *Oprk1* (pseudocolored yellow) mRNA expression in H_2_O (n = 6) and EtOH (n = 6) mice after TMT. (**H**) Pdyn (intensity/mm^2^), (**I**) pdyn (counts/mm^2^), and (**J**) Oprk1 (intensity/mm^2^) are shown. *p<0.05. **p<0.01.

Initial reports have identified the BNST as a mediator of stress responses to TMT in rats (Fendt et al., 2003); however, the role of KOR signaling in this process has not been explored. Thus, we next tested whether microinfusions of norBNI directly into the BNST would alter behavioral responses to TMT during protracted abstinence [Figure 3A–C, Figure 3—figure supplement 1]. Importantly, norBNI or PBS infusion into the BNST did not affect distance traveled during the TMT test [Figure 3D]. However, similar to systemic administration, intra-BNST norBNI reduced contact with TMT in the EtOH mice [Figure 3E; interaction F_1,35_=4.30, p=0.0454; PBS H_2_O vs EtOH t_35_ = 3.29, p=0.0105; EtOH PBS vs norBNI t_35_ = 3.32, p=0.0105] with no effect on time spent in the far corners of the home cage [Figure 3F]. EtOH mice showed significantly less burying behavior in response to TMT compared to H_2_O mice, but there was no effect of drug in EtOH mice [Figure 3G; EtOH main effect F_1,35_=42.65, p<0.001; PBS H_2_O vs EtOH t_35_ = 4.06, p=0.0010; norBNI H_2_O vs EtOH t_35_ = 5.19, p<0.001]. Intra-BNST norBNI did not alter behavior in the elevated plus maze [Figure 3H–I].

**Figure 3.** Role of BNST KOR in responses to predator odor after alcohol. (**A**) Experimental design for 5 µg/µl norBNI in the BNST. (**B**) Representative images of BNST infusions of PBS (n = 9 H_2_O, n = 10 EtOH) and norBNI (n = 10 H_2_O, n = 10 EtOH) marked with GFP. Scale bar indicates 200 µM. (**C**) Representative heatmaps of TMT-induced activity with EtOH BNST PBS (left) and EtOH BNST norBNI (right). (**D**) Distance traveled during the TMT test. (**E**) TMT contact (sec), (**F**), time spent in the far corners (sec), and (**G**), burying (sec) during the TMT trial. Time spent in the (**H**), open arms (sec) and (**I**) closed arms (sec) of the elevated plus maze. *p<0.05. **p<0.01.

**Figure 3—figure supplement 1.** Histological verification of stereotaxic injections in male mice. Correct placements of a single norBNI or PBS infusion are shown in coronal sections in millimeters from bregma surrounding the BNST of C57BL/6J mice. Circles represent the injection center of PBS, and crosses represent norBNI. Both groups had 10 nl GFP to mark the injection site.

We next examined the synaptic activity of BNST^PDYN^ neurons following TMT exposure by recording spontaneous excitatory and inhibitory post-synaptic currents (sEPSC, sIPSC) in Pdyn-GFP mice during 7–10 days protracted abstinence [Figure 4A]. TMT increased sEPSC frequency (Hz) in EtOH and H_2_O drinkers compared to non-stressed (NS) mice [Figure 4B; TMT main effect F_1,50_=18.24, p<0.0001; H_2_O NS vs TMT t_50_ = 3.38, p=0.0028; EtOH NS vs TMT t_50_ = 2.75, p=0.0167] with no alterations in sIPSC frequency [Figure 4C]. EtOH and TMT did not impact sEPSC and sIPSC amplitude [Figure 4—figure supplement 1A–B]. Increased sEPSC/sIPSC ratios also reflected heightened excitatory drive onto BNST^PDYN^ cells in stressed mice regardless of drinking history [Figure 4D; TMT main effect F_1,50_=23.61, p<0.0001; H_2_O NS vs TMT t_50_ = 2.50, p=0.0312; EtOH NS vs TMT t_50_ = 4.24, p=0.0002; TMT H_2_O vs EtOH t_50_ = 2.25, p=0.0566]. In the EtOH drinking, stressed group, there was a moderate correlation between cumulative EtOH drinking (g/kg) and sEPSC frequency [Figure 4—figure supplement 1C; R^2^ = 0.38, p=0.1062] and sEPSC/sIPSC ratio [Figure 4—figure supplement 1D; R^2^ = 0.31, p=0.1545]. We next examined if KOR played a role in driving this cellular phenotype. Systemic norBNI pretreatment reduced sEPSC frequency in BNST^PDYN^ cells [Figure 4E–F; norBNI main effect F_1,34_=7.94, p=0.008, EtOH TMT saline vs norBNI t_34_ = 3.22, p=0.0056], but not sIPSC frequency [Figure 4G], with an increase in the sEPSC/sIPSC ratio being suppressed by norBNI in the EtOH TMT mice [Figure 4H; norBNI main effect F_1,34_=9.36, p=0.0043; EtOH TMT saline vs norBNI t_34_ = 2.62, p=0.026]. NorBNI did not alter sEPSC or sIPSC amplitude in stressed mice [Figure 4—figure supplement 1E–F]. These ex vivo experiments demonstrate that exposure to stress and EtOH induces KOR-mediated alteration of synaptic transmission in the BNST.

**Figure 4.** KOR regulation of increased synaptic transmission onto BNST Pdyn neurons after stress and EtOH. (**A**) Representative traces of BNST^PDYN^ cell synaptic transmission in H_2_O (n = 6, 17 cells), EtOH (n = 4, 12 cells), H_2_O + TMT (n = 5, 15 cells), and EtOH + TMT (n = 4, 10 cells). Scale bar indicates 50 pA height and 1 s time. Spontaneous excitatory post-synaptic currents (sEPSC) are on the left, and spontaneous inhibitory post-synaptic currents (sIPSC) are on the right. (**B**) sEPSC frequency (Hz), (**C**) sIPSC frequency (Hz), and **D**), sEPSC/sIPSC ratio in dorsal BNST Pdyn cells. (**E**) Sample traces of BNST^PDYN^ cell synaptic transmission after 16 hr pretreatment with 5 mg/kg norBNI or saline, i.p. Aqua is saline + H2O + TMT (n = 4, 11 cells). Red is saline + EtOH + TMT (n = 4, 10 cells). Light aqua is norBNI + H_2_O + TMT (n = 3, 8 cells). Light red is norBNI + EtOH + TMT (n = 3, 9 cells). Scale bar equals 50 pA height and 1 s time. (**F**) sEPSC frequency (Hz). (**G**) sIPSC frequency (Hz). (**H**) sEPSC/sIPSC ratio. *p<0.05. **p<0.01.

**Figure 4—figure supplement 1.** Additional synaptic transmission elements of BNST Pdyn neurons after TMT stress and EtOH drinking. (**A**) TMT BNST^PDYN^ cell synaptic transmission sEPSC amplitude (pA). (**B**) sIPSC amplitude (pA). Correlation between cumulative, total EtOH (g/kg) across six weeks and (**C**) sEPSC frequency (Hz) and (**D**), sEPSC/sIPSC ratio in Pdyn-GFP mice after EtOH and TMT. (**E**) NorBNI pretreatment BNST^PDYN^ cell sEPSC amplitude (pA). (**F**) sIPSC amplitude (pA).

We then tested if dynorphin produced in the BNST played a role in behavioral changes following EtOH and TMT, as we have previously shown that BNST Pdyn can modulate synaptic transmission in the BNST (Crowley et al., 2016). *Pdyn* was deleted from the BNST using the *Pdyn^lox/lox^* mouse line (Bloodgood et al., 2020) via AAV Cre-GFP microinfusions [Figure 5A–B, Figure 5—figure supplement 1]. Pdyn deletion in the BNST did not alter EtOH consumption [Figure 5C–D; Time main effect F_17,323_=3.28, p=0.0095; Cumulative EtOH drinking (g/kg) per group: t_19_ = 0.23, p=0.8181] or preference [Figure 5E–F; Time main effect F_17,323_=4.09, p=0.0019; average EtOH preference per group: t_19_ = 0.10, p=0.9221]. EtOH history moderately augmented distance traveled in the TMT test [Figure 5H; EtOH main effect F_1,37_=6.20, p=0.0174], but Pdyn deletion was not a factor in this difference. EtOH mice with BNST Pdyn deletion suppressed EtOH-related increases in TMT contact [Figure 5G, Figure 5I; EtOH main effect F_1,37_=7.31, p=0.0103. GFP H_2_O vs EtOH t_37_ = 2.93, p=0.0347], and they increased their burying behavior compared to control EtOH mice [Figure 5K; interaction F_1,37_=4.51, p=0.0405. EtOH GFP vs EtOH Cre-GFP t_37_ = 3.91, p=0.0419]. Importantly, there were no effects of Pdyn deletion in H_2_O drinkers on TMT response, nor were there effects in the elevated plus maze [Figure 5L–M]. These findings demonstrate a role for BNST Pdyn/KOR in regulating specific behavioral responses impaired by long-term EtOH drinking.

**Figure 5.** EtOH drinking and TMT responses after BNST Pdyn deletion. (**A**) Time course of deletion of BNST Pdyn in *Pdyn^lox/lox^* mice before EtOH and TMT. (**B**) Images of AAV-GFP and AAV-Cre-GFP expression (H_2_O GFP n = 10, Cre-GFP n = 10. EtOH GFP n = 10, EtOH Cre-GFP n = 11). Scale bar measures 200 µM. (**C**) *Pdyn^lox/lox^* mice EtOH drinking (g/kg/24 hr) across 6 weeks with BNST GFP (red) or Cre-GFP (light red). (**D**) Cumulative EtOH drinking (g/kg) per group. (**E**) Average EtOH Preference ratio/24 hr per group across time. (**F**) Average EtOH Preference per mouse across the 6 weeks. (**J**) *Pdyn^lox/lox^* mice daily EtOH preference across 6 weeks with BNST GFP (red) or Cre-GFP (light red). (**K**) Average EtOH preference per group. (**G**) Sample TMT heatmaps of EtOH BNST GFP (left) and EtOH BNST Cre-GFP (right) mice. In the TMT test, (**H**) distance traveled (cm), (**I**) TMT contact, (**J**) far corners (sec), and (**K**) burying (sec). In the elevated plus maze, duration in the (**L**) open arms (sec), and (**M**) closed arms (sec). *p<0.05.

**Figure 5—figure supplement 1.** Histological verification of BNST Pdyn deletion. Correct BNST placements of AAV-Cre-GFP or AAV-GFP infusion are shown in coronal sections in millimeters from bregma in a floxed Pdyn mouse line. Injection centers are represented by circles for GFP or crosses for Cre-GFP.

Given that we have previously reported increased glutamatergic transmission in the mPFC following acute TMT exposure (Hwa et al., 2019) and recent reports from the Radley lab indicated a key role in PFC inputs to the BNST in stress regulation, we next wanted to investigate if EtOH and TMT together may strengthen the functional connection between mPFC and BNST Pdyn neurons. To do this, we injected an AAV encoding channelrhodopsin (ChR2) into the mPFC of Pdyn-GFP mice [Figure 6A] and measured BNST cell responses to photostimulation of this pathway using slice electrophysiology [Figure 6B]. A large proportion of BNST^PDYN^ neurons were light responsive after TMT in both H_2_O and EtOH mice, whereas non-stressed H_2_O mice had mostly non-responsive cells [Figure 6C; Χ^2^_3_ = 21.43, p<0.0001]. Similarly, EtOH mice had larger monosynaptic optically-evoked EPSC (oEPSC) amplitudes following TMT compared to H_2_O mice and non-stressed EtOH mice [Figure 6D; interaction F_1,33_=4.74, p=0.0367; H_2_O non-stress (NS) vs EtOH + TMT t_33_ = 3.70, p=0.0047; EtOH NS vs EtOH + TMT t_33_ = 4.50, p=0.0005], with no effects on paired pulse ratio [Figure 6E]. Both AMPA and NMDA peak amplitudes were greater in BNST^PDYN^ EtOH TMT mice compared to unstressed EtOH mice and H_2_O mice [Figure 6F–G; AMPA peak amplitude: TMT main effect F_1,34_=22.03, p<0.0001; H_2_O NS vs EtOH + TMT t_34_ = 4.28, p=0.0009; EtOH NS vs EtOH + TMT t_34_ = 4.82, p=0.0002. NMDA peak amplitude: TMT main effect F_1,34_=12.09, p=0.0148; H_2_O NS vs EtOH + TMT t_34_ = 3.13, p=0.0213; EtOH NS vs EtOH + TMT t_34_ = 3.27, p=0.0148]. There was also an increase in the AMPA/NMDA ratio in the EtOH TMT mice [Figure 6H; TMT main effect F_1,34_=8.12, p=0.0074; EtOH NS vs EtOH + TMT t_34_ = 2.89, p=0.0132], suggesting alcohol drinking may prime the synapse for AMPA receptor recruitment, further contributing to aberrant glutamate signaling and stress reactions. In addition, the EtOH TMT mice were also more resistant to synaptic depression of oEPSC amplitude in response to repeated 1 Hz oEPSC pulses, suggesting alterations in short-term plasticity [Figure 6I–L; interaction F_27,351_=1.83, p=0.0080; Pulse 3: EtOH NS vs EtOH + TMT t_22.81_=3.21, p=0.0234; H_2_O + TMT vs EtOH + TMT t_18.81_=3.40, p=0.0180; Pulse 4: EtOH NS vs EtOH + TMT t_23.99_=3.95, p=0.0036]. We next wanted to compare this mPFC-BNST pathway with another known glutamatergic input, so ChR2 was injected into the basolateral amygdala (BLA) in another group of Pdyn-GFP mice for slice recordings [Figure 6—figure supplement 1A]. The BLA input to the BNST is large, as most cells were responsive to photostimulation in all groups [Figure 6—figure supplement 1B]. In contrast to the mPFC-BNST pathway, EtOH drinking and TMT exposure did not affect BLA-BNST oEPSC amplitude [Figure 6—figure supplement 1C], paired pulse ratio [Figure 6—figure supplement 1D], AMPA peak amplitude [Figure 6—figure supplement 1E], NMDA peak amplitude [Figure 6—figure supplement 1F], or AMPA/NMDA ratio [Figure 6—figure supplement 1G]. There were also no major group differences in BLA-BNST oEPSCs in response to repeated pulse trains [Figure 6—figure supplement 1H–K].

**Figure 6.** Cortical input onto BNST^PDYN^ cells gates stress-enhanced glutamatergic plasticity after history of alcohol. (**A**) Image of CamKII-ChR2-mCherry expression in the mPFC (left) and at BNST terminals (right). Pdyn-GFP cells are green. Inset photo scale bars measure 100 µm. Representative traces of optically-evoked mPFC action potentials at 1 Hz. Blue rectangles indicate 470 nm LED onset. Scale bar indicates 20 mV and 1 s. (**B**) Experimental design testing synaptic connectivity of mPFC input to BNST^PDYN^ cells using channelrhodopsin (ChR2) after EtOH and TMT. (**C**) Proportions of light-responsive (white) and non-light-responsive (grey) BNST^PDYN^ cells to optically evoked EPSC in H_2_O (10/27 responsive cells, n = 7), EtOH (14/21 responsive cells, n = 5), H_2_O + TMT (9/11 responsive cells, n = 4), and EtOH + TMT (11/13 responsive cells, n = 4) groups. (**D**) mPFC-BNST^PDYN^ oEPSC amplitude (pA). (**E**) Paired pulse ratio. Inset example traces of H_2_O + TMT (aqua) and EtOH + TMT (red) with blue LED onset. Scale bar indicates 200 pA height and 50 ms time. (**F**) AMPA peak amplitude (pA). Inset AMPA traces of H_2_O + TMT (aqua) and EtOH + TMT (red) with blue LED onset. Scale bar indicates 200 pA height and 50 ms time. (**G**) NMDA peak amplitude (pA). Inset NMDA traces of H_2_O + TMT (aqua) and EtOH + TMT (red) with blue LED onset. Scale bar indicates 200 pA height and 50 ms time. (**H**) AMPA/NMDA ratio. (**I**) Representative traces of 1 Hz pulse trains in EtOH + TMT (red) and H_2_O + TMT (aqua) BNST^PDYN^ cells. Scale bar indicates 200 pA height and 1 s time. oEPSC normalized amplitude across (**J**) 1 Hz, (**K**) 5 Hz, and (**L**) 10 Hz pulse trains. *p<0.05. **p<0.01.

**Figure 6—figure supplement 1.** Basolateral amygdala input onto BNST^PDYN^ cells after history of alcohol and TMT exposure. (**A**) Experimental design testing synaptic connectivity of basolateral amygdala (BLA) input to BNST^PDYN^ cells using channelrhodopsin (ChR2) after EtOH and TMT. (**B**) Proportions of light-responsive (white) and non-light-responsive (grey) BNST^PDYN^ cells to optically-evoked EPSC in H_2_O (6/8 responsive cells, n = 3), EtOH (6/9 responsive cells, n = 4), H_2_O + TMT (14/14 responsive cells, n = 4), and EtOH + TMT (14/14 responsive cells, n = 4) groups. (**C**) BLA-BNST^PDYN^ oEPSC amplitude (pA). (**D**) Paired pulse ratio. Inset example traces of H_2_O + TMT (aqua) and EtOH + TMT (red) with blue LED onset. Scale bar indicates 500 pA height and 50 ms time. (**E**) AMPA peak amplitude (pA). Inset AMPA traces of H_2_O + TMT (aqua) and EtOH + TMT (red) with blue LED onset. Scale bar indicates 1000 pA height and 50 ms time. (**F**) NMDA peak amplitude (pA). Inset NMDA traces of H_2_O + TMT (aqua) and EtOH + TMT (red) with blue LED onset. Scale bar indicates 200 pA height and 500 ms time. (**G**) AMPA/NMDA ratio. (**H**) Representative traces of 1 Hz pulse trains in EtOH + TMT (red) and H_2_O + TMT (aqua) BNST^PDYN^ cells. Scale bar indicates 200 pA height and 1 s time. oEPSC normalized amplitude across (**I**) 1 Hz, (**J**) 5 Hz, and (**K**) 10 Hz pulse trains. *p<0.05.

To investigate the behavioral role of the PFC-BNST pathway in vivo, we performed pathway-specific chemogenetic manipulations with designer receptors exclusively activated by designer drugs (DREADDs). A retrograde AAV containing cre recombinase was injected into the BNST, and an AAV containing cre-inducible hM4Di-mCherry or mCherry was injected into the mPFC of C57BL/6J mice [Figure 7A–B; Figure 7—figure supplement 1]. Bath application of CNO on mPFC cell bodies infected with cre-inducible hM4Di-mCherry produced hyperpolarization of resting membrane potential [Figure 7C] and increased latency to fire action potentials [Figure 7D]. The inhibitory DREADD alone did not affect drinking behavior across the 6 weeks [Figure 7E] or short-term drinking behavior when CNO was injected versus saline [Figure 7F–H]. When exposed to TMT, hM4Di-mediated inhibition of the mPFC-BNST pathway did not alter distance traveled [Figure 7J], but it did reduce contact with TMT in both H_2_O and EtOH mice [Figure 7I, Figure 7K; virus main effect: F_1,25_=5.37, p=0.0289; no significant post-hoc differences]. Time spent in the far corners was not affected [Figure 7L]. mPFC-BNST inhibition also increased burying behavior in EtOH-drinking mice [Figure 7M; EtOH main effect: F_1,25_=13.80, p=0.001; virus main effect: F_1,25_=16.47, p=0.004; H_2_O mCherry vs EtOH mCherry t_25_ = 4.37, p=0.0234; EtOH mCherry vs EtOH hM4Di t_25_ = 4.72, p=0.0131]. Time spent in the open and closed arms of the elevated plus maze were also not affected by the inhibitory DREADD [Figure 7N–O].

**Figure 7.** DREADD-mediated inhibition of mPFC-BNST pathway and assessment of EtOH drinking and TMT-related behaviors. (**A**) Time course of mPFC-BNST chemogenetic strategy in C57BL/6J mice before EtOH and TMT. (**B**) Images of AAV-hM4Di-mCherry expression in mPFC cell bodies, left, and BNST terminals, right (H_2_O mCherry n = 7, H_2_O hM4Di-mCherry n = 7. EtOH mCherry n = 8, EtOH hM4Di-mCherry n = 7). mCherry was enhanced with a GFP immunostain. Slice physiology validation of the DREADD strategy, in mPFC neurons, as represented by (**C**), hyperpolarization of resting membrane potential after CNO bath application. Inset scale bar indicates 2 mV height and 30 s time. (**D**) Latency to action potential threshold before and after CNO with 100 pA current ramp steps. Scale bar indicates 20 pA height and 100 ms time. (**E**) EtOH drinking (g/kg/24 hr) across 6 weeks with mPFC-BNST hM4Di (red) or mCherry (light red). EtOH intake (g/kg) across (**F**) 1 hr, (**G**) 4 hr, and (**H**) 24 hr after i.p. saline (circles) or 3 mg/kg CNO (diamonds). (**I**) Sample TMT heatmaps of EtOH mPFC-BNST mCherry (left) and EtOH mPFC-BNST hM4Di (right) mice. In the TMT test, (**J**) distance traveled (cm), (**K**) TMT contact, (**L**), far corners (sec), and (**M**), burying (sec). In the elevated plus maze, duration in the (**N**), open arms (sec), and (**O**), closed arms (sec). *p<0.05.

**Figure 7—figure supplement 1.** Histological verification of multiplexed DREADD injection sites. (**A**) mPFC placements of AAV-DIO-hM4Di-mCherry or AAV-DIO-mCherry and, (**B**) BNST placements of retrograde AAV-Cre infusion are shown in coronal sections in millimeters from bregma in C57BL/6J mice. Injection centers are represented by circles for mCherry or crosses for hM4Di-mCherry.

## Discussion

Here, we have identified a causal role for the mPFC-BNST^PDYN^ pathway in mediating alcohol-induced alterations in TMT predator odor-evoked stress responses. First, we identified BNST^PDYN^ as a stress- and alcohol-sensitive population using immunohistochemistry and in situ hybridization. With whole cell patch clamp electrophysiology, we found that enhanced synaptic drive in BNST^PDYN^ cells was reduced by KOR antagonism in stressed mice with a history of alcohol drinking. Finally, experiments with ex vivo optogenetics indicated that EtOH-drinking stressed mice had increased prefrontal cortical synaptic connectivity onto BNST^PDYN^ cells compared to unstressed EtOH drinkers. We were able to manipulate EtOH-induced alterations in TMT stress reactions using BNST KOR antagonism, BNST Pdyn deletion, and PFC-BNST chemogenetic inhibition. Altogether, our findings indicate that engagement of Pdyn/KOR signaling in the BNST promotes an allostatic shift in stress-responses following EtOH drinking.

### BNST KOR/Pdyn gates stress reactions after EtOH

Previous articles from our laboratory have shown that wild-type and transgenic mice exhibit relatively modest intermittent EtOH drinking and preference (Bloodgood et al., 2020) compared to those reported in Hwa et al., 2011 publication, which was likely a results of varying vivarium conditions. However, mice in this study still achieved intoxicating blood EtOH concentrations, and this intermittent schedule may be favorable over drinking levels in continuous two-bottle choice access (Yu et al., 2019). In our hands, 6 weeks of intermittent access to EtOH affected behavioral responses to TMT predator odor. We interpret the EtOH-induced lack of avoidance of the predator odor as a maladaptive reaction to an innately stressful stimulus. While control mice displayed an array of stress behaviors in response to TMT (i.e. freezing, grooming, stretch-attend, etc.), a lack of burying was a prominent behavioral feature of EtOH mice. Burying in response to an immediate threat is commonly interpreted as an innate, active coping behavior in rodents (De Boer and Koolhaas, 2003).

While EtOH mice also showed increased anxiety-like behavior in the elevated plus maze during protracted withdrawal, this group difference was eliminated following TMT exposure, as seen in our control drug/virus experiments after BNST norBNI, Pdyn deletion, and mPFC-BNST inhibition, suggesting long-lasting impact of TMT on performance in the elevated plus maze (EPM). Since we chose to not use another cohort of surgerized/transgenic mice for testing in the EPM, it is important to note that testing without prior TMT exposure was a limitation. TMT can have mixed effects on time spent in the open arms of the EPM, which can be dependent on the TMT concentration (Hacquemand et al., 2013; McGregor et al., 2002; Makhijani et al., 2020). This points to the EPM as a distinct, novelty-related probe, which may not be robust to differentiate EtOH-related phenotypes after a confounding TMT exposure.

Using converging approaches of intra-BNST norBNI infusions and genetic deletion of BNST^PDYN^ using a floxed mouse line, we show that reducing Pdyn/KOR signaling at the pre- or post-synaptic level, respectively, normalizes alcohol-induced impairments in TMT behavioral responses during protracted abstinence. These results are in line with literature showing KOR antagonists can block anxiety-like behaviors precipitated by acute withdrawal from alcohol vapor (Valdez and Harshberger, 2012; Rose et al., 2016) and suppress alcohol self-administration in post-dependent rats (Walker and Koob, 2008; Schank et al., 2012; Kissler et al., 2014). KORs in the BNST appear to be particularly important in mediating interactions between stress and alcohol drinking, as BNST norBNI attenuates stress-induced alcohol seeking (Lê et al., 2018) and reduces alcohol withdrawal-induced 22 kHz ultrasonic vocalizations (Erikson et al., 2018). While this previous research has established that there is critical involvement of this stress peptide system in promoting acute alcohol withdrawal behaviors, we demonstrate here that KOR is still engaged in protracted abstinence, particularly during episodes of high stress exposure. Taken together, this body of evidence suggests that KOR signaling in the BNST is a critical pharmacological target for treatment of alcohol use disorders.

Our findings using c-Fos immunolabeling show that BNST^PDYN^ cells are synergistically engaged in responses to stressors in EtOH-drinking mice. This complements existing c-Fos work in the BNST after TMT predator odor exposure (Day et al., 2004; Asok et al., 2013; Janitzky et al., 2015) while newly connecting the Pdyn population with changes in stress responses following a history of EtOH drinking. As we were using a GFP reporter line to determine Pdyn-containing neurons, we also thought it was important to measure Pdyn and Oprk1 expression using fluorescence in situ hybridation. We observed that there was greater Pdyn content in EtOH mice, specifically a significant increase of Pdyn intensity and a trend towards Pdyn number. This suggests that increased c-Fos and Pdyn co-localization after EtOH exposure and stress could be due to the emergence of a larger pool of Pdyn neurons. Future studies should measure real-time engagement of BNST^PDYN^ neurons during TMT exposure using fiber photometry, as specific subpopulation of BNST neurons are known to exhibit TMT-elicited calcium transients (Giardino et al., 2018).

### Glutamatergic contribution to stress-enhanced signaling in BNST^PDYN^ neurons

After assessing population activity of BNST PDYN/KOR after EtOH and stress and the contributions of this population to drinking-induced alterations in behavior, we performed synaptic transmission experiments on BNST^PDYN^ neurons during protracted abstinence from EtOH. In addition, non-stressed intermittent EtOH mice displayed modestly increased sIPSC frequency in BNST^PDYN^ cells. While some studies from our laboratory have reported increased sIPSC frequency in the BNST 24 hr after drinking in monkeys (Pleil et al., 2015), others have found increased sEPSC/sIPSC ratios in C57BL/6J mice 48 hr after ethanol vapor (Pleil et al., 2016) These differences are likely the result of cell-type-specific population targeting, variations in drinking/exposure protocols, and withdrawal time points. During protracted abstinence, there were no apparent synaptic transmission differences between withdrawn mice and controls, although previous reports have found increased sEPSC frequency at this time point in female drinkers in a BNST CRF population (Centanni et al., 2019). Rather, we found that TMT exposure increased glutamatergic transmission in BNST^PDYN^ neurons after EtOH and TMT, suggesting enhanced glutamatergic activity across the region. While BNST^PDYN^ synaptic drive did not differ between stressed H_2_O and EtOH mice, differences in transmission were revealed during KOR blockade with norBNI pretreatment. Altogether, while other studies have found that chronic EtOH exposure and withdrawal can impact BNST spontaneous glutamatergic and NMDAR function (Kash et al., 2009; Wills et al., 2012; McElligott and Winder, 2009), our findings are the first to highlight plastic shifts in response to stressors and identify pathway-specific alterations in neuropeptide signaling.

### EtOH and stress interact revealing synaptic plasticity from cortical input

The mPFC, among other brain regions, is a known source of increased glutamatergic signaling onto BNST neurons. Previous work in the lab found that both central amygdala (CeA) and basolateral amygdala (BLA) inputs to the BNST are KOR-sensitive, but mPFC inputs are KOR-insensitive (Crowley et al., 2016). Notably, photostimulation of BLA inputs promotes anxiolysis in alcohol-naive mice (Crowley et al., 2016). Taken together, these findings suggest a model in which increased activity of BNST^PDYN^ neurons promote release of Pdyn, which in turn inhibit amygdala inputs to the BNST to promote increased engagement of mPFC glutamate signaling. We have previously identified prelimbic (PL) layer 2/3 neurons as a population engaged in response to acute TMT using a combination of slice physiology and immunohistochemical approaches (Hwa et al., 2019), providing converging data for engagement of this pathway by this specific aversive stimulus. However, while Pdyn/KOR signaling in the CeA appears to promote EtOH consumption (Bloodgood et al., 2020), Pdyn/KOR signaling in the BNST did not affect EtOH drinking in our study.

Our study provides valuable insight into how the synaptic strength of the mPFC to BNST^PDYN^ pathway may be altered by combined exposure to EtOH and stress. Indeed, we found that a higher proportion of BNST^PDYN^ neurons were light-responsive following stress or EtOH compared to H_2_O controls, suggesting that these stimuli increase connectivity between the mPFC and BNST^DYN^ neurons. Taking into account the observed increases in oEPSC, AMPA, and NMDA amplitudes and AMPA/NMDA ratio after the combination of EtOH and TMT, it appears that EtOH exposure primes the synapse for aberrant responses to stressors under the control of a glutamatergic, mPFC-driven mechanism. Further, with repeated stimulation pulse trains, the EtOH TMT BNST^PDYN^ cells show reduced short-term depression, suggesting increased fidelity and short-term plasticity in this circuit. Again, this is in line with known chronic EtOH-induced glutamate plasticity in BNST cells (Wills et al., 2012). In contrast to the mPFC-BNST pathway, we observed no differences in the strength of BLA inputs to BNST^PDYN^ neurons after EtOH and stress. Since there was a stress-EtOH interaction observed from the cortical projection, we wanted to examine how inhibition of this pathway could alter behavior. In an mPFC-BNST DREADD experiment, we found that chemogenetic inhibition also improved burying behavior in EtOH mice. This was specific to TMT behavior, as the manipulation did not affect EtOH drinking or anxiety-like behavior in the elevated plus maze. It is also possible that systemic CNO injection may impact behavior via effects on collaterals of those mPFC-BNST that project to other brain regions. This is a caveat, and intra-BNST delivery of CNO would be more direct. These combined strategies of testing synaptic strength in slice and pathway-specific manipulation of behavior provide a mechanism for how long-term drinking and stress interact to dysregulate prefrontal inputs to BNST^PDYN^ neurons.

### BNST circuitry control of stress behavior

A recent paper from the Radley lab explored the role of the PL mPFC to BNST pathway in stress-related behaviors in rats using optogenetics (Johnson et al., 2019). Activation of the PL to BNST circuit negatively correlated with freezing behavior, a measure of passive coping, in response to a shock prod, while photoinhibition increased freezing and decreased burying, a measure of active coping. Notably, they found that these behavioral effects were related to downstream control of the periaqueductal gray. An important future direction will be to assess the role of specific downstream projection targets of BNST Pdyn neurons, including the periaqueductal gray, in EtOH-induced alterations in TMT behavioral responses. It is also possible that excitatory local microcircuity in the BNST activates GABA neurons that inhibit ventral tegmental area GABA output signaling reward, which leads to anhedonia-like behavior and reduced stress responding. Our results illustrating aberrant responses to stress during protracted withdrawal from alcohol complement established research characterizing a more general role for the BNST in anxiety-related behaviors employing chemo- and optogenetics in mice (Kim et al., 2013; Jennings et al., 2013; Marcinkiewcz et al., 2016; Mazzone et al., 2018; Crowley et al., 2016).

### Conclusions

Maladaptive responses to stress are a hallmark of alcohol use disorder, but the mechanisms that underlie this effect are not well characterized. Here, we show that Pdyn/KOR signaling in the BNST is a critical molecular substrate disrupting stress-related behavioral responses following heavy alcohol drinking. Further, our findings suggest that increased corticolimbic connectivity may underlie this phenomenon; thus, altered mPFC-BNST connectivity could serve as a potential biomarker of negative outcomes in alcohol use disorder. Disentangling this imbalance of corticolimbic-driven stress neuropeptide signaling may lead to the development of novel therapeutics to enhance stress coping in persons with alcohol use disorder.

## Materials and methods

**Key resources table:** 

Reagent type (species) or resource	Designation	Source or reference	Identifiers	Additional information
Strain, strain background (*Mus musculus* male)	C57BL/6J	Jackson Laboratories	B6/J	Stock # 000664
Strain, strain background (*Mus musculus* male)	*Pdyn^IRES-Cre^*	Jackson Laboratories	B6;129S-*Pdyn^tm1.1(cre)Mjkr^*/LowlJ	Stock # 027958
Strain, strain background (*Mus musculus* male)	EGFP-*L10a*	Jackson Laboratories	B6;129S4-*Gt(ROSA) 26Sor^tm9(EGFP/Rpl10a)Amc^*/J	Stock # 024750
Strain, strain background (*Mus musculus* male)	*Pdyn^lox/lox^*	Bloodgood et al., 2020		
Antibody	anti-c-Fos (Rabbit polyclonal)	Millipore	Cat# ABE457, RRID:AB_2631318	(1:3000)
Antibody	anti-rabbit horse radish peroxidase-conjugated IgG (Goat polyclonal)	PerkinElmer	Cat# NEF812001EA, RRID:AB_2571640	(1:200)
Antibody	anti-mCherry (Chicken polyclonal)	Abcam	Cat# ab205402, RRID:AB_2722769	(1:500)
Antibody	Alexa Fluor 488 anti-chicken (Donkey polyclonal)	Jackson Immuno Research Laboratories	Cat# 703-545-155, RRID:AB_2340375	(1:200)
Strain, strain background (AAV)	AAV5-CamKII-Cre-eGFP	UNC Vector Core	Lot 6450	
Strain, strain background (AAV)	AAV5-CamKII-eGFP	UNC Vector Core	Lot 4621B	
Strain, strain background (AAV)	AAV5-CamKIIa-hChR2(H134R)-mCherry-WPRE-hGH	Addgene	Lot CS1096	
Strain, strain background (AAV)	AAV8-hSyn-DIO-hM4D(Gi)-mCherry	Addgene	Lot 6048	
Strain, strain background (AAV)	AAV2retro-SL1-CAG-Cre	Janelia	Custom Prep	
Sequence-based reagent	Mm-Oprk1	ACDbio	316111	
Sequence-based reagent	Mm-Pdyn	ACDbio	318771	
Commercial assay or kit	TSA amplification kit with Cy3	PerkinElmer	Cat# NEL744001KT	(1:50)
Commercial assay or kit	RNAscope Florescent Multiplex Assay	ACDbio		
Commercial assay or kit	Corticosterone ELISA Kit	Arbor Assays		
Chemical compound, drug	norBNI	Tocris	Cat# 0347	
Chemical compound, drug	CNO	Hello Bio	Cat# HB6149	
Software, algorithm	Prism 8	GraphPad		
Software, algorithm	ClampFit 10.7	Molecular Devices		
Software, algorithm	Ethovision XT	Noldus		
Software, algorithm	BORIS	Friard and Gamba	DOI:10.1111/2041-210X.12584	
Other	TMT	BioSRQ	Cat# 1G-TMT-97	
Other	Peanut oil	Harris Teeter		

### Animals

Eight-week-old male C57BL/6J mice (Jackson Laboratories, Bar Harbor, ME) were used for behavioral pharmacology experiments. To visualize Pdyn-expressing neurons, we generated a Pdyn-GFP reporter line by crossing *preprodynorphin*-IRES-Cre mice (Crowley et al., 2016; Bloodgood et al., 2020; Al-Hasani et al., 2015) (*Pdyn^IRES-Cre^*, B6;129S-*Pdyn^tm1.1(cre)Mjkr^*/LowlJ, Jackson Laboratories Stock # 027958) and Rosa26-flox-stop-L10a-EGFP reporter mice (EGFP-*L10a*; B6;129S4-*Gt(ROSA)26Sor^tm9(EGFP/Rpl10a)Amc^*/J, Jackson Laboratories Stock # 024750). For conditional knockout of BNST Pdyn, we used the *Pdyn^lox/lox^* mouse line (Bloodgood et al., 2020). These mice were bred in the UNC facilities. All mice were group-housed for at least 3 days before being singly housed in polycarbonate cages (GM500, Tecniplast, Italy) with a 12:12 hr reversed dark-light cycle with lights off at 7:00am. Mice had unrestricted access to food (Prolab Isopro RMH 3000, LabDiet, St. Louis, MO) and H_2_O. The UNC School of Medicine Institutional Animal Care and Use Committee approved all experiments. Procedures were conducted in accordance with the NIH Guidelines for the Care and Use of Laboratory Animals.

### Intermittent EtOH drinking

Mice were given 24 hr access to a 20% (w/v) EtOH solution and water on an intermittent schedule (Hwa et al., 2011). Two bottles were held in modified drinking spouts of plastic cage tops and weighed before and after daily EtOH access. A dummy cage without an animal was used to simulate fluid lost while positioning the bottles, so average fluid drip was subtracted from each mouse’s daily drinking. Mice were tested for stress reactions to TMT during 7–10 day protracted abstinence after 6 weeks of intermittent drinking. Blood EtOH concentrations were measured in a subset of mice. Tail blood was collected after 2 hr of intermittent EtOH drinking, and then centrifuged at 3000 rpm at 4°C. Separated blood plasma was stored at −20°C before analysis using the AM1 Analox Analyzer (Analox Intstruments Ltd., Lunenberg, MA).

### Behavioral assays after EtOH drinking

#### TMT predator odor exposure

Exposure to fox-derived synthetic predator odor, trimethylthiazoline (TMT), was performed in the home cage as previously described to elicit stress reactions in mice (Hwa et al., 2019). Animals were moved to a separate experimental room for testing that included a fume hood and a large fan. Mice were tested one at a time for odor removal between trials. The lid of the home cage was removed for videorecording. Tests were conducted under dim lighting conditions, 15–20 lux. For a baseline pre-trial period, mice habituated to a cotton tip applicator held vertically in place for 10 min in the home cage. The TMT trial occurred when 2.5 µl TMT was applied to the cotton tip followed by 10 min of behavioral observation. As a control odor, 2.5 µl peanut oil (Harris Teeter, Carrboro, NC) was applied to the cotton tip in a separate group of mice. Duration of contact with the TMT object, time spent in the far corners of the cage, and distance traveled (sec) were recorded and quantified with Ethovision XT13 (Noldus, The Netherlands). Heatmaps were generated through Ethovision XT13. Burying was hand-scored using BORIS (Behavioral Observation Research Interactive Software) by a blind observer. The BORIS software also generated representative ethograms/Gantt plots of stress-related and exploratory behaviors, including duration and frequency of burying, freezing, grooming, rearing, stretch-attend, and walking.

#### Plasma corticosterone assay

To measure plasma corticosterone 30 min following TMT predator odor exposure, 5 µl plasma samples were processed with a commercially available colorimetric ELISA kit (Arbor Assays, Ann Arbor, MI), according to the manufacturer’s instructions. All samples were run in duplicates.

#### Elevated plus maze

Mice were placed into the center of an elevated plus maze (75 cm) and allowed to explore for 5 min (Bloodgood et al., 2020; Crowley et al., 2016; Mazzone et al., 2018). Light levels in the open arms were approximately 15 lux. Duration of time spent in the open arms and closed arms were recorded and calculated by Ethovision XT13. The time interval between TMT and elevated plus maze tests was 3 days.

### Stereotaxic surgery

Adult mice (>8 weeks) were deeply anesthetized with 3–4% isoflurane in oxygen and placed into a stereotaxic frame (Kopf Instruments, Tujunga, CA) while on a heated pad. Isoflurane anesthesia was maintained at 1–2% during the remainder of the surgery. After sterilization with 70% ethanol and betadine, a scalp incision was made and burr holes were drilled above the target. A 1 µl Neuros Hamilton syringe (Hamilton, Reno, NV) microinjected the virus or drug at a rate of 0.1 µl/min. Coordinates for the dorsal BNST were AP +0.30 mm, ML +/- 0.95 mm, DV −4.35 mm from bregma. Coordinates for the mPFC were AP +1.70 mm, ML +/- 0.30 mm, DV −2.50 mm from bregma. Coordinates for the BLA were AP −1.30 mm, ML +/- 3.25 mm, DV −4.95 mm from bregma. Mice recovered for 1 week before testing.

### Drugs and viral vectors

5 mg/kg norBNI (Cat no. 0347, Tocris) or saline was administered i.p., 1 ml/100 g, 16 hr before testing to both EtOH and H_2_O mice. For intra-BNST norBNI microinfusions, 5 µg/µl norBNI or PBS was injected with 50 nl AAV5-CamKII-eGFP to mark the injection site. Intra-BNST administration of norBNI or PBS was a single, bilateral infusion of drug. Since animals underwent stereotaxic surgery for drug delivery, 7 days was the minimum time for post-operative recovery before TMT behavioral testing. Both 16 hr and 7 day drug pretreatment minimized handling stress prior to the predator odor exposure and allowed for KOR antagonism instead of non-specific mu opioid antagonism that occurs initially post-injection. norBNI is known for its ultra-long duration of action (Munro et al., 2012). While we did not directly test to see if KOR antagonism was still pharmacologically effective at the time of TMT and EPM testing, previous studies have shown the effects of norBNI in the mouse tail flick test up to 28 days after administration (Horan et al., 1993) and rat intracranial self-stimulation thresholds for at least 86 days after administration (Potter et al., 2011). Therefore, it is likely that norBNI was on board at the time of TMT testing.

*Pdyn^lox/lox^* mice received 300 nl AAV5-CamKII-Cre-eGFP (UNC Vector Core, Lot 6450) and control AAV5-CamKII-eGFP (Lot 4621B) in the BNST. 300 nl AAV5-CamKIIa-hChR2(H134R)-mCherry-WPRE-hGH (Addgene, Lot CS1096) was injected into the mPFC or BLA of Pdyn-GFP mice for synaptic connectivity experiments in the BNST. C57BL/6J mice were injected with 300 nl AAV8-hSyn-DIO-hM4D(Gi)-mCherry (Addgene, Lot 6048) into the mPFC and AAV2retro-SL1-CAG-Cre into the BNST for mPFC-BNST inhibition. All intracranial injections were bilateral.

To test DREADD-mediated inhibition on EtOH consumption, saline and CNO were administered 20 min before EtOH drinking on two final test days. EtOH and H_2_O fluid consumption were measured after 1, 4, and 24 hr. During protracted withdrawal 7 days later, CNO was administered 20 min before the TMT test, and again 20 min before testing in the EPM, which occurred after 3 days. 3 mg/kg clozapine N-oxide (CNO; Hello Bio, Princeton, NJ) was dissolved in saline before i.p. administration, 1 ml/100 g, 20 min before testing.

### c-Fos immunohistochemistry, histology, and microscopy

For c-Fos and histological verification, mice were deeply anesthetized with Avertin before transcardial perfusion with phosphate buffered saline and 4% paraformaldehyde. Brains were extracted 90 min following TMT exposure for c-Fos, cryoprotected, and then sliced at 45 µm on a Leica 1200S vibratome. Coronal sections of the Pdyn-GFP mice were stained for *c-Fos* immunofluorescence to visualize colocalization of Pdyn-containing (GFP) and *c-Fos* expressing cells. The immunofluorescence protocol for *c-Fos* was performed according to previous studies (Hwa et al., 2019) using tyramine signal amplification (TSA). After PBS washes, 50% methanol, and 3% hydrogen peroxide, tissue was incubated in blocking buffer with 0.3% Triton X-100% and 1% bovine serum albumin for 60 min. Slices were then incubated at 4°C for 48 hr in blocking buffer containing a rabbit anti-*c-Fos* antibody (1:3000, ABE457, Millipore, Bellerica, MA). After washes in TNT (0.1 M Tris-HCl, 0.15 M NaCl, 3% TritonX-100) and TNB (0.1 M Tris-HCl, 0.15 M NaCl, 0.5% Perkin Elmer blocking reagent) buffer, slices were incubated in a goat anti-rabbit horse radish peroxidase-conjugated IgG (1:200, NEF812001EA, PerkinElmer, Waltham, MA) for 30 min. After TNT washes, tissue was processed using a TSA kit with Cy3-tyramide (1:50, PerkinElmer, Waltham, MA) for 10 min. For the mPFC-BNST chemogenetic inhibition experiment, we enhanced the mCherry signal in the mPFC cell bodies and BNST terminals using a similar immunofluorescence protocol. After PBS washes, 3% hydrogen peroxide, PBS washes, and 30 min in 0.5% Triton X-100, tissue was incubated in 0.1% Triton X-100, 10% normal donkey serum, and 1% bovine serum albumin for 60 min. Slices were then incubated at 4°C for 24 hr in blocking buffer containing a chicken anti-mCherry antibody (1:500, ab205402, Abcam, Cambridge, MA). After PBS washes, tissue underwent secondary incubation for 2 hr at room temperature in PBS containing Alexa Fluor 488 donkey anti-chicken (1:200, Jackson ImmunoResearch Laboratories, Inc West Grove, PA).

For placement verification, viral injection sites were verified using a wide-field epifluorescent microscope (BX-43, Olympus, Waltham, MA). For quantification of *c-Fos* immunofluorescence, slices were imaged on a Zeiss 800 laser scanning confocal microscope (Carl Zeiss, Germany) and analyzed with Zeiss Zen 2 Blue Edition software. Using the Image Analysis Wizard in the Zen Blue software, Pdyn-GFP cells were identified as the parent classifier, and c-Fos Cy3-labeled cells were identified as the child classifer. Automatic segmentation parameters were identical for each image within each new frame drawn to delineate the dorsal BNST. Pdyn-GFP cells, c-Fos cells, and c-Fos cells nested within Pdyn-GFP cells were automatically counted for each image. Four coronal brain sections containing the bilateral BNST were stained, imaged, and analyzed for each animal.

For in situ hybridization, brains were extracted 30 min following TMT exposure under isoflurane anesthesia. Tissue was flash frozen on dry ice for 15 min and stored at −80°C until sectioned for in situ hybridization. 18 µm coronal slices containing the BNST were made on the Leica CM 3050S cryostat (Leica Biosystems, Nussloch, Germany) at −20°C, mounted directly onto microscope slides, and stored at −80°C. In situ was performed according to the manufacterer’s protocol for fresh frozen tissue sections (RNAscope Fluorescent Multiplex Assay; ACDbio, Newark, CA) with the following exceptions. PBS washes following tissue fixation were extended to 5 min each and protease treatment was shortened to 15 min. Probes utilized were RNAscope Probe-Mm-Oprk1 (Cat no 316111) and RNAscope Probe-Mm-Pdyn (Cat no 318771). Slides were incubated with DAPI, coverslipped with ProLong Gold (Life Technologies), and imaged on a Zeiss 800 laser scanning confocal microscope. ImageJ was used to count mean intensity of fluorescence for *Pdyn* (550 channel) and *Oprk* (647 channel), and the cell counter plug-in was used to hand count Pdyn-positive neurons. After verification with DAPI, cells labeled with at least three puncta were counted as containing Pdyn mRNA. Hand counts were tabulated by a blind observer.

### Slice electrophysiology

Ninety minutes following TMT, during 7–10 day protracted withdrawal, mice were sacrificed via deep isoflurane anesthesia, and coronal brain slices containing the BNST were collected according to standard laboratory protocols (Hwa et al., 2019; Crowley et al., 2016; Bloodgood et al., 2020). Whole-cell voltage-clamp electrophysiological recordings were performed in dorsal BNST^PDYN^ cells. Pdyn-GFP-containing cells were selected based on visualization using a 470 nm LED and GFP filter. The effects of EtOH and TMT on basal synaptic transmission were assessed in voltage clamp by adjusting the membrane potential and using a cesium methanesulfonate-based intracellular solution (135 mM cesium methanesulfonate, 10 mM KCl, 10 mM HEPES, 1 mM MgCl2, 0.2 mM EGTA, 4 mM MgATP, 0.3 mM GTP, 20 mM phosphocreatine, pH 7.3, 285–290 mOsmol). Lidocaine n-ethyl bromide (1 mg/ml) was included in the intracellular solution to block postsynaptic sodium currents. Neurons were held at −55 mV to assess glutamatergic synaptic transmission. In the same cell, neurons were held at +10 mV to assess GABAergic synaptic transmission. Fluctuations in current were used to determine spontaneous post-synaptic current (sEPSC or sIPSC) frequency and amplitude, as well as to calculate sEPSC/sIPSC ratios. Synaptic transmission experiments in BNST^PDYN^ cells were also performed in animals that received 5 mg/kg norBNI i.p. 16 hr prior to TMT. Electrophysiological recordings were then analyzed using Clampfit 10.7 software (Molecular Devices, Sunnyvale, CA).

For ex-vivo optogenetic experiments, tissue was evaluated for light-evoked action potentials in the mPFC. Brains were discarded and not used for further experimentation if injection sites were missed or if action potentials were not present. A blue LED (470 nm, CoolLed) was used to optically stimulate release from channelrhodopsin (ChR2)-containing fibers (Crowley et al., 2016). Picrotoxin (25 μM), tetrodotoxin (500 nM), and 4-AP (200 μM) were added to the aCSF to isolate monosynaptic oEPSCs with cells held at −70 mV. The intracellular solution was cesium gluconate (117 mM D-gluconic acid and cesium hydroxide, 20 mM HEPES, 0.4 mM EGTA, 5 mM tetraethyl ammonium chloride, 2 mM MgCl26H2O, 4 mM Na2ATP, 0.4 Na2GTP, pH 7.3, 287–292 mOsmol). oEPSC amplitude (pA) was the first peak of the paired pulse ratio with a 50 ms interstimulus interval. Paired pulse ratio was calculated as the second peak amplitude divided by the first peak amplitude. Cells were held at −70 mV to isolate AMPAR-mediated current and at +40 mV for NMDAR-mediated current. In separate slices, ten 1, 5, and 10 Hz pulse trains were performed at −55 mV voltage clamp without the presence of ionotropic inhibitors with the cesium methanesulfonate internal solution. The nine subsequent amplitudes in the pulse train were normalized to the first peak.

For DREADD validation in slice, mPFC cell bodies were identified with mCherry expression. 10 µM CNO (Hello Bio, Princeton, NJ) was bath applied for 10 min, and the resting membrane potential was monitored in voltage clamp. Action potential firing was assessed before and after CNO application using an increasing ramp protocol in current clamp.

### Statistics

Time spent in contact with the TMT, far corners, and burying behavior in seconds (s), and distance traveled (cm) were analyzed with two-way ANOVA with drug/virus and EtOH as factors. Post-hoc paired and unpaired t-tests were two-tailed and used where appropriate. In experiments where virus was injected before EtOH, cumulative 6 week alcohol intake and average ethanol preference were compared via t-test. BNST *c-Fos*, Pdyn-containing, and *c-Fos* and Pdyn colocalization were analyzed with two-way ANOVA with TMT exposure and EtOH as factors. With norBNI physiology, saline- and norBNI-injected stressed mice were compared in separate two-way ANOVA with drug and EtOH as factors. To compare proportion of light-responsive cells per condition, a Χ^2^ test was performed. Furthermore, optically-evoked experiments (e.g. oEPSC amplitude) were analyzed with two-way ANOVAs comparing TMT and EtOH exposure. Pulse trains were analyzed with repeated measures two-way ANOVA across stimulus time and condition. Alpha was set to 0.05. Biological replicates throughout behavioral, immunohistochemical, and electrophysiological studies were combined. Statistical tests were analyzed with GraphPad Prism 8 (La Jolla, CA, USA).

## Data Availability

All data are available in the main text or the supplementary materials.

## Additional files

Transparent reporting form
